The article "Circular RNA hsa_circ_0072309 inhibits non-small cell lung cancer progression by sponging miR-580-3p" was retracted in 2021. Reasons: duplicated images; original data or images not available.

# Circular RNA hsa_circ_0072309 inhibits non-small cell lung cancer progression by sponging miR-580-3p

**DOI:** 10.1042/BSR20194237

**Published:** 2020-05-04

**Authors:** Wenguang Pang, Fengliu Huang, Xin Zhang, Min Ye, Yanming Huang, Xiufang Huang, Jingzhuo Pang, Chengjie Cai, Zheng Wang

**Affiliations:** 1 Department of Thoracic Surgery, The First Affiliated Hospital of Jinan University, Guangzhou 510630, China; 2 Department of Thoracic Surgery, Jiangmen Central Hospital, Jiangmen 529030, China; 3 Department of Respiration Medicine, Jiangmen Central Hospital, Jiangmen 529030, China; 4 Clinical Experimental Center (Clinical Biobanks), Jiangmen Central Hospital, Jiangmen 529030, China; 5 Department of Pathology, Jiangmen Central Hospital, Jiangmen 529030, China; 6 Department of Thoracic Surgery, The 2nd Clinical Medical College of Jinan University, Shenzhen 518020, China

**Keywords:** hsa_circ_0072309, miR-580-3p, non-small cell lung cancer

## Abstract

**Objective:** Non-small cell lung cancer (NSCLC) continues to top the list of cancer mortalities worldwide. Early diagnosis and therapeutic interventions targeting NSCLC is becoming the world’s significant challenge. Circular RNAs (circRNAs) are emerging as a group of potential cancer biomarkers.

**Materials and methods:** Quantitative real-time PCR (qRT-PCR) was employed to examine the expression of circ_0072309 in NSCLC tissues and cell lines. Cell counting kit 8 (CCK-8), wound healing and Transwell assays were used to analyze cell proliferation, migration and invasion in A549 and H1299 cells. The relationship between circ_0072309 and miR-580-3 was analyzed by Luciferase reporter and RNA pull down assays.

**Results:** We screened circ_0072309 from Gene Expression Omnibus and found that circ_0072309 was lowly expressed in NSCLC tissues and cell lines. The transfection of circ_0072309-overexpressing vector significantly suppressed the cell proliferation, migration and invasion in A549 and H1299 cells. We predicted that miR-580-3p is a target of circ_0072309 by using publicly available bioinformatic algorithms Circinteractome tool and confirmed that circ_0072309 directly bound to miR-580-3p. Furthermore, the addition of miR-580-3p mitigated the blockage of cell proliferation, migration and invasion induced by circ_0072309.

**Conclusions:** These data showed that circ_0072309 inhibits the progression of NSCLC progression via blocking the expression of miR-580-3p. These findings revealed the anti-tumor role of circ_0072309 during the development of NSCLC and provided a novel diagnostic biomarker and potential therapy for NSCLC.

## Introduction

Lung cancer is one of the most commonly found carcinoma type and is an aggressive tumor with high incidence and mortality rate worldwide [1]. Non-small cell lung cancer (NSCLC) accounts for 80–85% of lung cancer diagnoses and is the major cause of lung cancer-associated mortality due to late-stage detection [2]. Despite advances in clinical and experimental oncology have been made in recent years, the 5-year overall survival rate of NSCLC is still limited [3]. Thus, to explore the molecular mechanisms of NSCLC and to identify effective biomarkers is essential for NSCLC early diagnosis and treatments.

The article "Circular RNA hsa_circ_0072309 inhibits non-small cell lung cancer progression by sponging miR-580-3p" was retracted in 2021. Reasons: duplicated images; original data or images not available.

Circular RNAs (circRNAs) are a new class of noncoding RNA molecules with the length of at least a few hundred nucleotides lacking 5′ caps or 3′ poly-A tails [4]. CircRNAs are reported to closely associate with the progression of a large number of cancers [5]. Aberrant regulation of circRNAs has been noted in gliomas [6], renal cell carcinomas [7] and other human malignancies [8]. With the development of high-throughput sequencing and bioinformatics analysis, increasing numbers of novel circRNAs have been identified to be potential cancer prognostic biomarkers [9]. CircRNA has_circ_0072309 was identified to be located on chromosome 5 between the base sites 38523520 and 38530768 [10]. Some reports showed that has_circ_0072309 was lowly expressed in breast cancer [11,12], human intracranial aneurysms [10] and renal carcinoma [13]. However, the function of has_circ_0072309 in the progression of NSCLC remains elusive.

In the present study, we screened the circ_0072309 from GSE112214 dataset. Quantitative real-time PCR (qRT-PCR) results showed that circ_0072309 was down-regulated in NSCLC tissues and cell lines. The overexpression of circ_0072309 significantly blocked the cell proliferation, migration and invasion in A549 and H1299 cells. Luciferase reporter and RNA pull down assays indicated that circ_0072309 directly bound to miR-580-3p. The blockage of cell proliferation, migration and invasion induced by circ_0072309 was mitigated by miR-580-3p mimic. Taken together, our study indicated that circ_0072309 blocks NSCLC tumor progression by sponging miR-580-3p. These findings provided a novel biomarker and potential treatment strategy for NSCLC diagnosis and clinical treatment.

## Materials and methods

### Clinical samples

The clinical specimens including 30 pairs of NSCLC tissues and adjacent normal tissues were isolated from patients who underwent surgery between 2016 and 2018 at the Department of Thoracic Surgery, The 2nd Clinical Medical College of Jinan University. Patients did not receive any preoperative therapy, including radiotherapy and chemotherapy before surgery. The pathological diagnosis of tissue samples were performed by two pathologists according to WHO grade criteria. All tissues were isolated and immediately transferred into liquid nitrogen for follow-up experiments. All patients have signed the informed consents prior to their participation in the study. The study was reviewed and approved by the Ethics Committee of The 2nd Clinical Medical College of Jinan University.

The article "Circular RNA hsa_circ_0072309 inhibits non-small cell lung cancer progression by sponging miR-580-3p" was retracted in 2021. Reasons: duplicated images; original data or images not available.

### Cell culture and transfection

Normal human bronchial epithelial cell line (HBE, BNCC338600) and four human NSCLC cells lines including CALU3 (BNCC338499), H125 (BNCC100831), A549 (BNCC100258) and H1299 (BNCC100268) were purchased from BeNa Culture Collection (Beijing, China). Cells were maintained in Roswell Park Memorial Institute-1640 (RPMI-1640, Invitrogen, Thermo Fisher Scientific, Waltham, MA, U.S.A.) containing 10% fetal bovine serum (FBS, Gibco, Grand Island, NY, U.S.A.) under the atmosphere containing 5% CO_2_ at 37°C.

Circ_0072309 was inserted into the pcDNA3.1 vector (pcDNA3.1-circ_0072309) to construct circ_0072309-overexpressing vector. For circ_0072309 overexpression, cells were transfected with pcDNA3.1-circ_0072309 (circ_0072309) or empty pcDNA3.1 (Vector). The miR-580-3p mimic and miR-NC were purchased from GenePharma (Shanghai, China). The transfections were performed using Lipofectamine 3000 (Invitrogen, Carlsbad, CA, U.S.A.) according to the manufacturer’s instructions. After 48 h, cells were collected for follow-up experiments.

### qRT-PCR

Total RNA was extracted from tissues or cells by using TRIzol (Invitrogen, Carlsbad, CA, U.S.A.) according to the manufacturer’s protocol. The cDNA was synthesized with First Strand cDNA Synthesis Kit (TaKaRa, Dalian, Liaoning, China). SYBR Premix ExTaq II Kit (TaKaRa, Dalian, Liaoning, China) was used to determine the expression level of target genes through the StepOnePlus system (Applied Biosystems, CA, U.S.A.) in line with the manufacturer’s protocol, and the 2^−ΔΔ*C*_T_^ method was adopted to calculate the relative expression of circ_0072309 and miR-580-3p. The primers for qRT-PCR were listed as follows: circ_0072309 forward primer (F): 5′- ggtcccgttcttgttagact-3′, reverse primer (R): 5′-gatggtcgtttcaaacatac-3′; miR-580-3p F: 5′-gccgagttgagaatgatgaa-3′, R: 5′-tggtgtcgtggagtcgg-3′; GAPDH F: 5′-gggaaactgtggcgtgat-3′, GAPDH R: 5′-gagtgggtgtcgctgttga-3′; U6 F: 5′-ctcgcttcggcagcaca-3′, R: 5′-aacgcttcacgaatttgcgt-3′.

### Cell viability assay

Cell viability was determined by using cell counting kit 8 (CCK-8, Donjindo, Kumamoto, Japan). Cells were seeded into a 96-well plate at the density of 2 × 10^3^ cells/well. After 0, 24, 48, 72 and 96 h, cells were incubated with 10 μl of CCK-8 reagent and incubated at 37°C for 2 h. Finally, the optical density was measured using EnSpire™ 2300 Multilabel Reader (PerkinElmer Inc., Waltham, MA, U.S.A.) at the wavelength of 450 nm. The experiment was repeated three times independently.

The article "Circular RNA hsa_circ_0072309 inhibits non-small cell lung cancer progression by sponging miR-580-3p" was retracted in 2021. Reasons: duplicated images; original data or images not available.

### Wound-healing assay

Cells were seeded into a six-well plate until they reached 70–80% confluence as a monolayer. The cell monolayer was gently and slowly scratched with sterile plastic 20 μl micropipette tips across the center of the attached cells. After 0 and 24 h, images were captured using a light microscope (Olympus IX81, Tokyo, Japan). The migration distance of the cells was measured using Image Pro-Plus version 6.0 (Media Cybernetics Inc., Rockville, MD, U.S.A.). The experiment was repeated three times independently.

### Transwell assay

Matrigel-coated (BD Biosciences, Franklin Lakes, NJ, U.S.A.) Transwell inserts (Costar, Manassas, VA, U.S.A.) were used to measure the invasive capacity of cells. The inserts were coated with 50 μl of 1 mg/ml Matrigel according to the manufacturer’s protocol. A total of 2 × 10^5^ cells in 200 μl of Dulbecco’s modified Eagle’s medium (DMEM) without serum were plated to the upper chamber. DMEM with 10% FBS was added to the lower compartment as a chemoattractant. After 24-h incubation, cells invading the lower surface of the membrane were fixed with cold methanol-glacial acetic acid and stained with 1% Crystal Violet for 15 min at room temperature. For each membrane, five fields (up, down, center, left and right, ×200) were selected for cell counting and photographed under the microscope (Canon, Tokyo, Japan). Transwell assays were performed with two technical replicates and three independent biological replicates.

### Biotinylated-RNA pull down

Biotinylated miR-580-3p probe was synthesized by GenePharma (Shanghai, China). Cells were seeded into six-well plates and transfected with bio-miR-580-3p or bio-miR NC at a final concentration of 20 nM for 24 h. The probe was incubated with M280 streptavidin dynabeads (Life Technologies Inc., Rockville, Maryland, U.S.A.) at 25°C for 2 h to generate probe-coated beads. The biotin–conjugated RNA complex was pulled down after incubation of the cell lysates with streptavidin-coated magnetic beads and extracted with TRIzol reagent. The level of circ_0072309 in bound fractions was evaluated by qRT-PCR analysis.

### Luciferase report assay

The luciferase reporter plasmid (Luc) was purchased from OBiO Technology (Shanghai, China). Sequences containing potential wild-type or mutant binding sites for miRNAs in circ_0072309 were cloned downstream of the luciferase gene promoter (Luc-circ_0072309 or Luc-circ_0072309-mutant). Cells were seeded into 24-well plates at the concentration of 5 × 10^4^ cells/well and co-transfected with Luc-circ_0072309 or Luc-circ_0072309-mutant, with miR-580-3p mimic or miRNA NC. After 48 h, cells were extracted and the Dual Luciferase Reporter Assay was measured using the dual-luciferase reporter assay system (Promega, Madison, WI, U.S.A.) by normalizing the firefly luminescence to *Renilla* luminescence. The experiment was repeated three times independently.

The article "Circular RNA hsa_circ_0072309 inhibits non-small cell lung cancer progression by sponging miR-580-3p" was retracted in 2021. Reasons: duplicated images; original data or images not available.

### Statistical analysis

Data were presented as the mean ± standard deviation. Statistical analysis was carried out with IBM SPSS version 18.0 (SPSS, Inc., Chicago, IL, U.S.A.). Difference between two groups was analyzed using Student’s *t* test and the analysis of multiple groups was carried out by using one-way analysis of variance followed by Dunnett’s post-hoc analysis. *P<0.05 was considered to indicate a statistically significant difference. All experiments in the present study were repeated three times at least.

## Results

### Circ_0072309 is down-regulated in NSCLC tissues and cell lines

We analyzed the microarray data (GSE112214 containing three pairs of NSCLC tissues and matched non-tumor tissues) from the GEO database (http://www.ncbi.nlm.nih.gov/gds/). The criteria for selection of differentially expressed circRNAs were |log2FC (fold change)| ≥ 1 and *P*<0.05. The top 15 up- and 15 down-expressed circRNAs were displayed in Figure 1A by using heatmaps. We found that the expression of circ_0072309 in NSCLC tissues was the lowest. In addition, in GSE112214 dataset, the expression of circ_0072309 in three NSCLC tissues was lower than that in matched non-tumor tissues (Figure 1B). We further collected 30 patients and confirmed the expression of circ_0072309 in NSCLC tissues and non-tumor tissues in Figure 1C. Similar results observed that circ_0072309 was down-regulated in patient-derived NSCLC tumor specimens versus adjacent healthy lung tissues. We extended our analysis from NSCLC tumor tissues to NSCLC cell lines. Compared with HBE, the expression of circ_0072309 in NSCLC cell lines (CALU3, H125, A549 and H1299) was significantly blocked (Figure 1D). Among the four NSCLC cell lines, circ_0072309 expression in A549 and H1299 cells was lower than that in CALU3 and H125 cells. We selected A549 and H1299 cells for subsequent cir_0072309 overexpression experiments. Taken together, these data indicated that circ_0072309 is poorly expressed in NSCLC tissues and cell lines.

**Figure 1:** circ_0072309 is poorly expressed in NSCLC tissues and cell lines (**A**) The heatmaps displayed the top 15 up- and down-expressed circRNAs between NSCLC and adjacent non-tumor tissues in GSE112214 based on the criteria of |log2FC| > 1 and *P*<0.05. Red in the two plots denoted up-regulation and blue stood for down-regulation. (**B**) circ_0072309 was lowly expressed in three NSCLC tissues in comparison with adjacent non-tumor tissues in GSE112214 dataset. (**C**) circ_0072309 was down-regulated in patient-derived NSCLC tumor specimens versus adjacent healthy lung tissues (*n*=30). (**D**) The expression of circ_0072309 was blocked in NSCLC cell lines. Total RNA was extracted from tissues or cells and qRT-PCR was performed to detect the expression of targets. **P<0.01.

The article "Circular RNA hsa_circ_0072309 inhibits non-small cell lung cancer progression by sponging miR-580-3p" was retracted in 2021. Reasons: duplicated images; original data or images not available.

### circ_0072309 inhibits cell proliferation, migration and invasion in A549 and H1299 cells

To explore the role of circ_0072309 in NSCLC carcinogenesis, we transfected A549 and H1299 cells with pcDNA3.1-circ_0072309 and empty pcDNA3.1 (Vector), and then performed CCK-8, wound-healing and Transwell assays. qRT-PCR was employed to confirm the transfection efficiency. In Figure 2A, compared with Vector group, the transfection of pcDNA3.1-circ_0072309 significantly enhanced the expression of circ_0072309, suggesting that pcDNA3.1-circ_0072309 was successfully overexpressed in A549 and H1299 cells. In Figure 2B, CCK-8 assay results showed that circ_0072309 overexpression significantly inhibited A549 and H1299 cell viability compared with that in Vector-transfected cells. These data showed that circ_0072309 inhibited cell proliferation in NSCLC cells.

**Figure 2:** The overexpression of circ_0072309 significantly blocks cell proliferation, migration and invasion (**A**) The transfection of pcDNA3.1-circ_0072309 up-regulated the expression of circ_0072309 determined by qRT-PCR in A549 and H1299 cells. (**B**–**D**) The overexpression of circ_0072309 blocked the cell viability, migration and invasion determined by CCK-8, wound healing and Transwell assays in A549 and H1299 cells. Cells were transfected with pcDNA3.1-circ_0072309 (circ_0072309) or pcDNA3.1 (vector). Total RNA was extracted for qRT-PCR and cells were collected for CCK-8, wound healing and Transwell assays. **P<0.01.

We further examined the effect of circ_0072309 on migration and invasion capabilities through wound healing and Transwell assays. In Figure 2C, compared with the Vector group, cells transfected with pcDNA3.1-circ_0072309 showed a wider wound area at 24 h after cell propagation. Similarly, the overexpression of circ_0072309 significantly decreased the number of invasive cells compared with Vector group in Figure 2D. These results showed that circ_0072309 prevented cell migration and invasion in NSCLC cells. Taken together, the overexpression of circ_0072309 significantly blocks cell proliferation, migration and invasion in A549 and H1299 cells.

The article "Circular RNA hsa_circ_0072309 inhibits non-small cell lung cancer progression by sponging miR-580-3p" was retracted in 2021. Reasons: duplicated images; original data or images not available.

### circ_0072309 serves as a sponge for miR-580-3p

To determine the mechanism of circ_0072309 functioning in NSCLC, we first analyzed the subcellular location of circ_0072309 by qRT-PCR and found that circ_0072309 was mainly located in the cytoplasm shown in Figure 3A. Many circRNAs may act as competitive endogenous RNAs and modulators of miRNA activity by competing for miRNA-binding sites [14]. Based on the prediction provided by publicly available bioinformatics algorithms Circinteractome tool (https://circinteractome.nia.nih.gov), we fortunately found a putative miR-580-3p binding site on the circ_0072309 sequence. To explore the relationship between circ_0072309 and miR-580-3p, we first constructed a wild-type (circ_0072309 wt) or a mutant (circ_0072309 mut) luciferase reporter plasmid (Figure 3B). Cells co-transfected with circ_0072309 wt and miR-580-3p mimic significantly decreased the luciferase signal in comparison with cells transfected with circ_0072309 wt and miR NC (Figure 3C). However, no significant difference was detected in the luciferase signal intensity of circ_0072309 mut between the miR-580-3p mimic and miR NC (*P*>0.05). These findings indicated that circ_0072309 bound to miR-580-3p. We further performed an RNA pull down using a biotin-labeled miR-580-3p probe. In Figure 3D, circ_0072309 was enriched within the miR-580-3p probe pull-down RNA complex in comparison with miR NC. These data suggested that circ_0072309 directly interacted with miR-580-3p. In A549 and H1299 cells, the overexpression of circ_0072309 significantly blocked the expression of miR-580-3p (Figure 3E), indicating that the negative relationship between circ_0072309 and miR-580-3p. Taken together, these data indicated that circ_0072309 serves as a sponge for miR-580-3p in A549 and H1299 cells.

**Figure 3:** circ_0072309 directly binds to miR-580-3p (**A**) circ_0072309 was localized at cytoplasm determined by qRT-PCR. (**B**) A wild-type (circ_0072309 wt) or a mutant (circ_0072309 mut) luciferase reporter plasmid was constructed based on the prediction by Circinteractome tool (https://circinteractome.nia.nih.gov). (**C**) Luciferase report assay was performed with circ_0072309 wt or circ_0072309 mut and miR-580-3p mimic. (**D**) RNA pull down was carried out with biotin-labeled miR-580-3p probe. (**E**) The overexpression of circ_0072309 significantly blocked the expression of miR-580-3p. (**F**) TCGA data showed that miR-580-3p was highly expressed in NSCLC tissues. (**G**) miR-580-3p was highly expressed in patient-derived NSCLC tumor specimens (*n*=30). **P<0.01. Abbreviation: TCGA, The Cancer Genome Atlas.

### circ_0072309 blocks cell proliferation, migration and invasion through miR-580-3p in NSCLC cells

After confirming the interaction between circ_0072309 and miR-580-3p, we further examined whether the anti-tumor function of circ_0072309 is attributed to its repression of miR-580-3p. We downloaded the data from The Cancer Genome Atlas (TCGA, https://cancergenome.nih.gov/). A total of 565 samples were included in the present study, containing 519 NSCLC samples and 46 matched non-tumor tissues. The expression of miR-580-3p in NSCLC tissues were significantly up-regulated than those in non-tumor tissues (Figure 3F). The similar trend was found in the patient-derived NSCLC tumor specimens versus adjacent healthy lung tissue (Figure 3G). These data suggested that miR-580-3p might exert as an oncogene in NSCLC progression. We transfected miR-580-3p mimic in circ_0072309-overexpressing cells and performed functional assays in Figure 4A. CCK-8 assay results showed that the overexpression of circ_0072309 significantly blocked cell viability, however, the addition of miR-580-3p mimic rescued the blockage of cell viability (Figure 4B). Similar results were observed in wound healing and Transwell assays. The administration of miR-580-3p mimic mitigated the blockage of the migration and invasion induced by circ_0072309 (Figure 4C,D). These data showed that the transfection of miR-580-3p mimic into circ_0072309 overexpressing cells rescued proliferation, migration and invasion defects, suggesting that circ_0072309 inhibited NSCLC progression through blocking the function of miR-580-3p.

The article "Circular RNA hsa_circ_0072309 inhibits non-small cell lung cancer progression by sponging miR-580-3p" was retracted in 2021. Reasons: duplicated images; original data or images not available.

**Figure 4:** The addition of miR-580-3p mimic rescues the blockage of cell proliferation, migration and invasion caused by circ_0072309 (**A**) The transfection of miR-580-3p mimic promoted the expression of miR-580-3p blocked by circ_0072309. (**B–D**) The addition of miR-580-3p mimic rescues the inhibition of cell proliferation, migration and invasion caused by circ_0072309 overexpression determined by CCK-8, wound healing and Transwell assays. Cells were randomly divided into three groups: Vector, circ_0072309 and circ_0072309+miR-580-3p mimic. Cells in circ_0072309 or circ_0072309+miR-580-3p mimic were transfected with pcDNA3.1-circ_0072309 or pcDNA3.1-circ_0072309+miR-580-3p mimic for 48 h, respectively. Vector group was transfected with pcDNA3.1. Cells were collected for CCK-8, wound healing and Transwell assays. **P<0.01.

## Discussion

Lung cancer is an aggressive tumor with high incidence and mortality rate [15]. NSCLC is responsible for poor survival of a majority of lung cancer patients [16]. Due to non-specific symptoms and no effectual diagnostic tests, approximately 70% of NSCLC are diagnosed at an advanced stage [17]. Non-invasive prognostic biomarkers are needed for the diagnosis of the advanced NSCLC patients with different histological types [18]. With the advance in the study of the molecular basis about lung cancer progression, targeted therapies have been used for NSCLC treatment [19].

The article "Circular RNA hsa_circ_0072309 inhibits non-small cell lung cancer progression by sponging miR-580-3p" was retracted in 2021. Reasons: duplicated images; original data or images not available.

CircRNAs are a group of non-coding RNAs with a stable closed-loop structure which prevents them from decomposing by the enzymes [20]. Increasing evidence indicated that circRNAs are closely associated with the progression of NSCLC [21]. For example, inhibition of circRNA VANGL1 suppresses the progression of bladder cancer [22]. Circ_000984 promotes cell proliferation and metastasis in NSCLC by modulating Wnt/β-catenin pathway [23]. CircRNA circFOXO3 promotes the prostate cancer progression [24]. The down-regulation of circRNA ciRS-7 [25] or circ_0067934 [26] blocks cell proliferation, migration and invasion of NSCLC cells. In our study, we found circ_0072309 was down-regulated in NSCLC tissues and cells, and the overexpression of circ_0072309 significantly blocked cell proliferation, migration and invasion, suggesting that circ_0072309 serves as a tumor suppressor in NSCLC. These data provided new evidence about the role of circRNA during the progression of cancers and provided a new biomarker for NSCLC diagnosis and therapy.

Emerging evidence showed that circRNAs were involved in the progression of tumors by acting as miRNA sponges in the cytoplasm [27], thereby regulating gene expression in transcriptional and post-transcriptional manners [28]. Previous study showed that circ_0072309 inhibits the proliferation and invasion in breast cancer via targeting miR-492 [12]. In human intracranial aneurysms, circ_0072309 acts as a ceRNA to affect discoid domain receptor 2 and systemic amino acid transporter 2 through miR-519e-5p and miR-516b-5p [10]. In renal carcinoma, circ_0072309 exerts anti-tumor roles by sponging miR-100 [13]. In our present study, we predicted that miR-580-3p is a target of circ_0072309 by bioinformatics analysis and employed luciferase report assay and RNA pull down methods to confirm that circ_0072309 directly binds to miR-580-3p. These data provided new evidence that miR-380-3p is a new target of circ_0072309 in NSCLC.

TWIST1 contributes to metastasis by promoting epithelial–mesenchymal transition and is misregulated in various cancers [29]. In breast cancer, miR-580 is able to target the 3′UTR of TWIST1 and overexpression of miR-580 inhibits cell motility [30]. It is reported that overexpression of miR-580 inhibits tumor growth in osteosaroma cell and the expression levels of miR-580 decreased with advanced tumor grade in glioma [31]. In neuroblastoma, serum miR-580 level is significantly up-regulated, which can be a potential prognostic marker [32]. miR-580 is identified to be positively associated with the pathogenesis and development of melanoma [33]. Although the role of miR-580 is reported, unfortunately, the knowledge of the function of miR-580-3p is very limited, especially their contribution to cancer progression. In our study, we found that miR-580-3p was highly expressed in NSCLC tissues, suggesting miR-580-3p was involved in the progression of NSCLC. In addition, the administration of miR-580-3p rescued the blockage of cell proliferation, migration and invasion induced by circ_0072309. These results further confirmed the role of circ_0072309 and miR-580-3p and revealed the mechanism that circ_0072309 inhibits the development of NSCLC by sponging miR-580-3p.

The article "Circular RNA hsa_circ_0072309 inhibits non-small cell lung cancer progression by sponging miR-580-3p" was retracted in 2021. Reasons: duplicated images; original data or images not available.

In summary, circ_0072309 blocks the progression of NSCLC by directly binding to miR-580-3p. These findings indicated that circ_0072309 could constitute a predictive biomarker and potential treatment strategy for NSCLC diagnosis and therapy.

## Abbreviations

CCK-8: cell counting kit 8
circRNA: circular RNA
DMEM: Dulbecco’s modified Eagle’s medium
FBS: fetal bovine serum
FOXO3: forkhead box O3
GAPDH: glyceraldehyde-3-phosphate dehydrogenase
GEO: gene Expression Omnibus
HBE: human bronchial epithelial
NSCLC: non-small cell lung cancer
qRT-PCR: quantitative real-time PCR
TWIST1: twist homolog 1
VANGL1: Vang-Like 1
